# Recent Techniques in Determining the Effects of Climate Change on Depressive Patients: A Systematic Review

**DOI:** 10.1155/2022/1803401

**Published:** 2022-08-08

**Authors:** Nur Izzati Ab Kader, Umi Kalsom Yusof, Mohd Nor Akmal Khalid, Nik Rosmawati Nik Husain

**Affiliations:** ^1^School of Computer Sciences, Universiti Sains Malaysia, Gelugor 11800, Penang, Malaysia; ^2^School of Information Science, Japan Advance Institute of Science and Technology, 1-1 Asahidai, Nomi 923-1292, Ishikawa, Japan; ^3^Department of Community Medicine, School of Medical Sciences, Universiti Sains Malaysia, Kota Bharu 16150, Kelantan, Malaysia

## Abstract

Climate change is amongst the most serious issues nowadays. Climate change has become a concern for the scientific community as it could affect human health. Researchers have found that climate change potentially impacts human mental health, especially among depressive patients. However, the relationship is still unclear and needs further investigation. The purpose of this systematic review is to systematically evaluate the evidence of the association between climate change effects on depressive patients, investigate the effects of environmental exposure related to climate change on mental health outcomes for depressive patients, analyze the current technique used to determine the relationship, and provide the guidance for future research. Articles were identified by searching specified keywords in six electronic databases (Google Scholar, PubMed, Scopus, Springer, ScienceDirect, and IEEE Digital Library) from 2012 until 2021. Initially, 1823 articles were assessed based on inclusion criteria. After being analyzed, only 15 studies fit the eligibility criteria. The result from included studies showed that there appears to be strong evidence of the association of environmental exposure related to climate change in depressive patients. Temperature and air pollution are consistently associated with increased hospital admission of depressive patients; age and gender became the most frequently considered vulnerability factors. However, the current evidence is limited, and the output finding between each study is still varied and does not achieve a reasonable and mature conclusion regarding the relationship between the variables. Therefore, more evidence is needed in this domain study. Some variables might have complex patterns, and hard to identify the relationship. Thus, technique used to analyze the relationship should be strengthened to identify the relevant relationship.

## 1. Introduction

Human health is acknowledged to be threatened by the climate change effects [1]. The term “climate” refers to the average of weather conditions in a particular region on Earth in terms of temperature, rainfall, and wind conditions based on historical data. The term “climate change” refers to long-term changes in the ordinary environment or climate instability [2]. Besides, climate change was defined by [3] as a shift in global or regional climate patterns, the most notable one is observable in the mid-to-late-twentieth century and is ascribed to the increase in carbon dioxide levels in the atmosphere as a result of the usage of fossil fuels.

Climate change is no longer a looming menace but a devastating fact with bleak future predictions [4]. While referring to the Intergovernmental Panel on Climate Change (IPCC) report in 2018 [5], the average global temperatures are continuing to rise in a more “stepped” manner than in previous years. Due to anthropogenic pollution, the average global temperature has increased by 0.6°C and is projected to increase. These events of global warming cause events such as the melting of ice caps, the submergence of coastal areas, adverse weather events, rainfalls, floods and droughts, wildfires in various regions, all likely to be linked to such gradual temperature rise [6, 7].

The climate change effects on vulnerable society and biological organisms concern the scientific community [8]. People are worried about climate change because it can have devastating consequences for the environment. It has been recognized as a critical global challenge, mainly when human activities have contributed to global climate [9]. The increased greenhouse effect causes “global warming,” or a rise in the Earth's surface temperature, over time. Temperature rise, changes in rainfall patterns, droughts, hurricanes, floods, and heatwaves, are forms of climate change [10]. Climate change effects on a global scale are expected to have a wide range of consequences for humanity. Climate change is understood to impact human health, both physical and mental. It is likely to be linked to the spread of vector-borne diseases, deaths and injuries caused by extreme weather, for example, flooding, hurricanes, and cyclones, thermal damage from exposure to heat, the likelihood of waterborne infection spread due to floods and coastal water warming, and a decrease in regional crop yields, all of which contribute to malnutrition. Climate change is predicted to have a substantial impact on human health [11].

While the physical health consequences of climate change are well established in the literature and practice, current research indicates that climate change and its associated weather events and environmental changes can substantially affect psychological well-being and mental health. The implications on mental health are among the lesser-known and frequently underestimated effects of climate change [12]. Recently, the temperature rise has been linked to an increase in mental illness problems, according to the research [13]. In parallel with an increasing consequence of climate change, mental illness problems have accounted for 13% of the global burden of disease. According to the World Health Organization (WHO), a mental disease is one of the leading causes of disability worldwide [14]. In low- and middle-income populations, the proportion of patients living with impairment due to mental disorders was 25.3% and 33.5%, respectively [15]. It could have a detrimental effect on public health, economic growth, and overall well-being. According to [13], current epidemiological connections between mental illness and environmental factors are increasingly being investigated, especially depression.

Depressive disorder or depression is one of the most common types of mental illness. It has grown into a significant public health issue. The number prevalence of depression globally increased from 172 million in 1990 to 258 million in 2017 [16]. It is reported that in 2020, more than 264 million people will be affected by depression worldwide [17]. Depression is severely impairing individuals' everyday functioning and quality of life and significantly contributing to global disability [18]. It is found that adolescents with severe depression are 30 times more likely to commit suicide [19]. Depression is also a significant cause of the almost 800,000 suicide fatalities every year [20]. Therefore, the burden of depression is a significant worry worldwide, particularly in low- and middle-income countries (LMIC)s. According to [21], the prevalence of depression is linked to substantial economic consequences with expensive healthcare costs. The cost of psychiatric disorders is among the challenges of healthcare policy. According to Lancet Psychiatry research, the total cost of treatment for depressive disorder (including anxiety) in 36 countries worldwide is expected to be 147 billion by 2030 [22]. It is the severe mental illness that should be paid attention to.

Previously, some researchers conducted reviews on the effects of climate change on a mental health such as [4, 8, 23–25]. Review by [4, 23] published in 2018 presents an overview of the hazards and impacts of climate change on mental health, both current and predicted. On the other hand, the remaining three reviews published in 2020 and 2021 also focus on summarising the evidence based on the epidemiological evidence on the effects of climate change on mental health. However, these review studies generally cover the climate change effects on overall mental health.

Therefore, this review narrows the scope only to consider the climate change effects on depressive disorder. The method of review study is based on the systematic literature review (SLR). Compared to other study review methods such as thematic, critical, or traditional narrative review, SLR implements a more thorough and well-defined evaluation process by adhering to procedures that involve exhaustive searches across all potentially significant studies, ensuring its replication by the provision of scientifically valid and open documentation of all research activity [26]. This is the first systematic review of climate change effects that focuses on depression to the best of our knowledge. The rationale for focusing only on depression is to obtain a more detailed insight by focusing only on the specific mental illness instead of general mental illnesses. It is critical to identify current literature gaps and establish future research objectives. This systematic review aims to systematically evaluate the evidence of the association between climate change effects on depressive patients. This systematic review may provide concrete evidence that can aid policymakers and clinicians in creating effective strategies to control and reduce the negative impacts of climate change on depressive patients.

Besides, based on the preliminary study, the researchers used different techniques such as correlation and time series analysis to determine the climate change effects on depression patients. Therefore, the technique is associated with correlation and time series in this systematic literature evaluation to acquire more precise results. The approaches related to the techniques will be identified using the search strategy. The review is conducted in accordance with the Preferred Reporting Items for Systematic Reviews and Meta-Analyses (PRISMA) standard. This systematic review aims to answer the following questions: 1. is there any association between environmental exposure related to climate change and mental health outcomes for depressive patients? 2. What are the techniques conducted for determining the climate change effects on depressive patients?

### 1.1. Objectives

The objectives of this systematic review were to:

1. Investigate the effects of environmental exposure related to climate change on mental health outcomes for depressive patients.
2. Analyzed the technique used to determine the relationship between climate change effects on depressive patients.
3. Identify the potential gaps and recommendations for future research.

## 2. Methods

A systematic review of the literature is a method for locating, selecting, and critically evaluating all relevant research and collecting and analyzing data from the studies included in the review. PRISMA guidelines were used for this review study. Based on [27] the advantage of PRISMA included (1) establishing a research question that allows for methodical research, (2) acknowledging the systematic review's inclusion and exclusion criteria, (3) aiming to look through an extensive database of scientific publications in a set amount of time.

### 2.1. Search Strategy

A well-planned and organized search strategy in an SLR is critical to ensure that all relevant work is discovered in the research results. As a result, a thorough search for relevant research articles was conducted to answer the research questions [28]. A comprehensive search strategy searched for studies in six electronic databases (Google Scholar, PubMed, Scopus, Springer, Science Direct, and IEEE Digital Library) from 2012 to September 2021. These six online databases were selected because they were considered the most appropriate databases that were providing comprehensive information related to the topic. The keywords employed in the study's search procedure were identified in the first step. Based on earlier studies and thesaurus, many terms comparable and linked to research topics were utilized for each online database. The keywords were: ((“effect” OR “impact” OR “consequence” OR “relationship” OR “association”) AND (“climate change” OR “global warming” OR “weather variability” OR “hot temperature” OR “heat”) AND (“depression” OR “depressive disorder” OR “distress”) AND (“correlation” OR “time series” OR “regression”)).

### 2.2. Inclusion and Exclusion Criteria

Some inclusion and exclusion criteria were established. Studies were considered for the evaluation if they explicitly assessed the effect of climate change on depressive patients and met the following criteria. Non-English publications were also omitted to avoid any misunderstandings about translated literature. In terms of timing, ten years (between 2012 and 2021) were chosen as sufficient time to comprehend the evolution of research and associated publications. Studies must be available in full text to obtain complete information. The article in terms of literature type like review articles, book series, novels, and book chapters were not included. As the review focuses on climate change effects on depression, articles not focused on depression are not considered.

### 2.3. Study Selection

Initially, 1823 articles were identified using specified keywords in electronic databases (Google Scholar, PubMed, Scopus, Springer, Science Direct, and IEEE Digital Library) with a range set from 2012 to 2021. The duplicated records were then removed. The first round of record screening was carried out to screen the articles based on their titles and abstracts. The articles that were entirely not related to inclusion criteria were removed. Next, the papers' full texts were reviewed and checked for eligibility criteria in the final stage. After investigation, only 15 studies were found to meet all the requirements for analysis.

### 2.4. Data Extraction

Data extraction was then performed to analyze the selected articles and dig out beneficial information using the data extraction form created in Microsoft Excel. Among the data extracted were the year of publication, author, environmental exposure, mental health outcome, vulnerability factors, the technique used in the study, and the type of work. The variables used should be related to the aim and objectives of this systematic review study.

### 2.5. Data Synthesis

The outcome from the data extraction was tabulated and synthesized in the narrative can be found in Section 3. Mostly, the finding was summarized based on the aim and objectives and research questions of this study.

## 3. Results

### 3.1. Study Identification

Finding the relevant articles in SLR is a long but systematic process.  Figure 1 shows the PRISMA flow diagram, which covers all stages in this review. Overall, 1823 papers were found, 1518 articles through Scopus, 62 through PubMed, 107 through Springer, 10 through Science Direct, 115 through Google Scholar, and 11 through IEEE Explore. After removing eight duplicate and 1735 unrelated articles, only 80 full-text articles were assessed for eligibility. The exclusion criterion excluded sixty-five articles after full-text reading. Finally, only 15 studies were included for analysis.

### 3.2. Characteristics of Included Study

The characteristics of the studies included are shown in Table 1. The study duration varied among the analyzed articles, ranging between 1 and 15 years. The most frequent study duration was 5 years [30–32]. The selected studies described the relationship between environmental exposure towards mental health outcomes of depressive patients in different ways. Two studies found a positive association between temperature and the increasing number of admissions of depressive patients [30, 31], with adjusted R-square, which was 56.58% (*p* < 0.001) and related risk (RR = 1.05) (1.01–1.09), respectively. One study reported a positive association between monthly hours of sunshine and frequency of admissions of depressive patients [33].

Another study, [36] found a correlation between temperature, atmospheric pressure, ozone and depression symptoms based on analyzed questionnaire responses. According to a study conducted in Ireland, participants who live in places with higher rainfall levels in preceding as well as current calendar months reported having more symptoms of depression (0.04 SE 0.02; *p*=0.039 for every 10 mm additional monthly rainfall), while participants who lived in the sunnier region reported having fewer depressive symptoms (−2.67 SE 0.88; *p*=0.003 for every additional hour of average annual daily sunshine) [34].

Three studies reported a positive association between air pollution and depression. [42] in their study reported a significant association between particulate matter pollution (PM) and depression, with the conclusion that PM exposure might become a crucial trigger for mental disease hospitalization, including depression. According to [43], ozone exposure was found to increase the rate of emergency admissions for depression in females 1–7 days after exposure and in males 1–5, and 8 days after exposure, with odds ratios ranging from 1.02 to 1.03. On the other hand, [44] reported a positive association between traffic-related air pollution (*PM*_10_, black carbon, *NO*_2_) and high odds of depressive disorder.

Two studies also found that drought duration was associated with high distress level [40, 41]. The study by [35] found no significant correlation between heat and humidity towards depression. Three studies reported that both low and high temperatures could increase the risk of depression. References [32, 37–39] reported that distinct climatic factors and seasons had a different impact on the hospital admission of depressive patients in the analyzed regions.

The selected articles also can be understood based on three aspects of the study: environmental exposure, mental health outcomes, and vulnerability factors. These three aspects also have been mentioned by [24] in their review.

### 3.3. Environmental Exposure

Environmental exposure means the type of climate change examined in the research, such as temperature (heat), humidity, rainfall, floods, drought, and wildfire. Regarding environmental exposure concerning depression, the researchers frequently considered temperature variables, followed by hours of sunshine, humidity, and air pollution. The other variables considered were drought, rainfall, duration of days, atmospheric pressure, and wind speed. However, these variables were infrequent compared to other variables. In the research, usually, researchers consider more than one variable except [32, 33, 37, 40, 41], and [43] that only focus on one variable for their research.

### 3.4. Mental Health Outcome

The mental health outcome measures the effects of the environmental exposure, such as hospital admissions, mortality, symptom scales, screening tools, and self-harm. The studies that utilize hospital admission as mental health outcomes routinely collected administrative data [45–48]. From the mental health outcome perspective used to measure those environmental exposures to depression, hospital admission is the most considered variable, followed by symptom scales and emergency department visits to verify the depression morbidity. Only one study measured the effects based on emergency department visit [43]. Besides, most of the studies [35, 40, 41, 44] measured the symptom based on the Kessler 10 (K10) Psychological Distress Index except two studies [34, 36]. The Kessler-10 is a brief assessment of general psychological discomfort comprised of questions about anxiousness, agitation, psychological exhaustion, and depression. It was created to be used on a scale ranging from mild to severe distress. Data were collected using a survey in most studies. The sample size varied from 1325 to 53,144 people.

### 3.5. Vulnerability Factors

Specific circumstances that may make people more susceptible to the mental health effects of climate change mean the vulnerability factors that might play a role in defining the link between environmental exposure and mental health outcomes, such as age, race, income. These factors are usually differently used between each study depending on the study's objectives. The vulnerability factors used in the selected studies are varied. Most of the variables were based on demographics, and the most frequently considered were age and gender. According to the [31], men with ages below 40 years are more susceptible to the impact of climate change. Reference [33] reported that the effects are different for males and females, where they found a significant increase in hospital admission for males aged greater than 65 and females aged (18–35) with greater amounts of sunlight. Reference [37] discovered that the elderly were more susceptible to the negative effects of heat exposure. In the elderly, males were more responsive to heat than females (HR = 1.18 vs 1.14). On the other hand, the younger group exhibited the reverse pattern (i.e., females 1.07 and males 1.04). In another research, males had higher associations with PM pollution and hospital admission than females, especially in cool seasons, according to [37]. Reference [34] in their research, specify the age group only to adults with 50 years and above, while [35] specify the age group as 45 years and above. Other factors included residency, employment status, history of mental health, educational level, relationship status, personal income, season, and insurance amount. However, they were not so frequently reported.

### 3.6. Study Techniques

Based on the selected studies, two categories of techniques were used to determine the climate change effects on depression: time series approaches and correlation analysis. All studies could be classified as using the time series approach except [36] which used correlation analysis.

Time series approach is a sequence of numbers, with the date and time stamps for recording those figures. Usually, the data is collected at regular intervals, such as an hour, day, month, or year. Time series is generally divided into time series analysis and time series forecasting. These two domains are closely related, but they perform differently: time series analysis is concerned with defining the intrinsic structure of time series data and interpreting the hidden traits to extract useful information (such as patterns or seasonal variance). Time series forecasting involves machine learning/deep learning models, training them using historical time-series data, and consuming them to forecast future predictions [49].

Time-series analysis is used to determine the effect of time-varying exogenous variables on a result over time [50]. As a result, the residual dependency must be assessed after the model has been fitted and modified for time-varying explanatory variables. Data scientists frequently use time series analysis for the following reasons: (i) develop a thorough understanding of the structural underpinnings of historical time series data. (ii) Increase the consistency of time series function interpretation to more effectively educate the problem domain. (iii) To enable a more lucrative and comprehensive historical data collecting, preprocessing, and feature engineering of high quality.

In environmental health investigations, standard time series analysis entails adjusting for unmeasured confounding variables such as long-term time patterns and seasons, air pollution, and influenza outbreaks [51]. In studies of the short-term effects of environmental stressors such as temperature on health outcomes, the following unmeasured time components are adjusted for: between-year trends; within-year trends (seasons); daily variability is left unadjusted but adjusted for other potential confounders that vary from the day today. Calendar patterns, such as weekdays and national holidays, are examples of such short-term possible confounding variables [50]. Estimating the variance in incident counts associated with ambient temperatures on the same day and preceding days (so-called lagged effects) is a typical objective of public health research, as there are frequently delays between exposure and effect [48].

The two most well-known methods of the techniques outlined above are statistics and machine learning. The statistical technique is a time-honoured model that has been in use for a very long period. Statistics are used to describe and infer data. Inferential statistics have been used to address data-related questions, test hypotheses (discovering and analyzing alternative or null hypotheses), generate an estimation of effect, typically a ratio of rates or risks, characterize associations (correlations) or model relationships (regression) within the data, and for a variety of other purposes. Point estimates are commonly used to assess the strength of relationships or the magnitude of impacts [52].

For statistical analysis, the researchers used regression models such as the stepwise regression model, log-linear function, linear regression model, logistic regression model, multivariable regression model, generalized additive model, Cox proportional hazard model, and autoregressive integrated moving average (ARIMA). The Pearson's correlation technique also has been applied to investigate the relationship between the variables.

Any data analysis procedure is designed to produce reasonable estimations from raw data. The statistical relationship between the response variable (Y) and the explanatory variables is commonly questioned (Xi). The link can be modelled using regression analysis. Regression analysis is available in a variety of configurations. If the distribution of Y is continuous and approximately normal, use linear regression; if the distribution is dichotomous, use logistic regression; if the distribution is Poisson or multinomial, use log-linear analysis; and if the distribution of Y is time-to-event, use log-linear analysis. Cox regression is used to forecast time-to-event data in cases that have been censored (survival-type data). The objective is to forecast the outcome (Y) using mathematical modelling based on the values of a set of predictor factors (Xi) [52].

Other than statistical analysis, the machine learning technique was also adopted in the study. In researching climate change effects on depressive disorder, the machine learning technique is relatively unexplored compared to the statistical approach. As of now, there is only one research that applied machine learning techniques for examining the impact of climate change on depressive patients. Reference [36] have used machine learning techniques in their research to identify the relationship between weather conditions and depression by using random forest and support vector machine after performing the correlation analysis.

The machine learning's aim is to create computer systems that can learn and adapt as a result of their experiences [53]. Machine learning is commonly used in intelligent systems with artificial intelligence capabilities today. Machine learning is the ability of a system to learn from problem-specific training data in order to automate the process of developing analytical models and completing associated tasks [54].

Also, correlation analysis is a commonly used statistical measure to find interesting collinear relations among different attributes of datasets. Pearson's correlation is one of the correlation analyses that previous researchers have applied to see the relationship between climate change and depression. This technique usually determines the relationship by a decimal value correlation coefficient. The strength and direction between the variables can be determined based on the value of the coefficient. It can help to find which independent variables have a significant impact on the dependent variable [55].

The coefficient value could be in the range of -1 to 1, with a maximum of 1. If the correlation coefficient value was positive, then there was a positive correlation; conversely, if the correlation coefficient value was negative, there would have been a negative correlation and vice versa. Reference [36] used this technique to investigate the association between temperature and other environmental exposure and mental health outcomes measured via symptom measures in a laboratory setting.

## 4. Comprehensive Science Mapping Analysis

The application of bibliometrics is getting popular in a variety of sectors. This technique is suitable in scientific mapping at a time when a strong emphasis on empirical evidence has resulted in multiple, fragmented, and controversial research streams [56, 57]. The article considered in this study was selected from six databases as elaborated in the study selection subsection, where most of the selected papers were based on the Scopus database with 83.27%. As mentioned previously, the category of study techniques in this review can be divided into statistical and machine learning techniques.  Figure 2 shows the percentage of articles based on each category. Most of the articles are based on statistical analysis. In terms of authorship, the majority of papers were collaborative research with many authors, with the exception of one study with a single author [39].

### 4.1. Most Relevant Sources

The distribution based on the most relevant sources based on the selected articles in this journal is shown in Table 2. The selected papers were retrieved from 12 different journals. None of the selected papers was published by conferences—the journals mostly related to environmental, public health, and psychiatry based on the result. The journals with the highest count of papers are Environmental Research, Science of The Total Environment, and Journal of Affective Disorders.

### 4.2. Annual Publication Production

The analysis of total selected papers (*n* = 15) based on annual publication production is shown in Figure 3. 2016 and 2021 were the year with the highest number of publications. No related publication was identified in 2013 and 2017. Nevertheless, it is worth mentioning that the topic interest is increasing, especially with the increasing trend in 2021. It is subsequent to the current prevalence of depressive disorder increasing in worrying trends nowadays.

### 4.3. Country-Wise Production

The publications based on country-wise production are shown in Figure 4. From the result, the highest number of publications was identified by Australian scholars, followed by China and Korea. The remaining countries were Canada, Belgium, Egypt, Vietnam, Poland, Ireland, Taiwan, and Iran, identified with a relatively equal number of published articles.

### 4.4. Word Cloud

A word cloud is a visual representation of the most significant topics associated with a particular subject [58].  Figure 5 presented the visualization of the keywords used in the selected articles in this study through the word cloud. Based on the word cloud visualization, the authors use a few of the most frequent keywords, such as hospital admission, depression, mental health, temperature, and climate. The larger the keyword's size in the cloud, the more frequently it was used in the studies.

## 5. Discussion

This section covers the analysis of results reported in Section 3. This SLR aims to systematically evaluate the evidence of the association between climate change effects on depressive patients, which investigates the effects of environmental exposure related to climate change on mental health outcomes for depressive patients, analyzing the current technique used to determine the relationship achieved. Most of the research was quantitative to determine the depressive hazards linked with climate change-related exposures.

A majority of selected literature indicates a positive association between environmental exposure and climate-change-related events and depression, except for a few studies that showed no significant association and inconsistency [35]. Climate-change-related events have been linked to an increase in the number of admissions, the frequency of admissions, the severity of depressive symptoms, and the level of distress experienced by depressive patients, and may serve as a critical trigger for mental disease hospitalizations including depression. However, it can be observed that the research investigating the impact of climate change on depression is still limited and needs more evidence in this area of study. In addition, the output finding of each study is still varied and does not achieve a reasonable and mature conclusion regarding the relationship between the variables. For example, the study from [35] found that a negative association between humidity towards depression is contrasted to the previous finding from [30]. Therefore, more evidence is needed to contribute toward a conclusive finding.

Additionally, selecting the relevant factors is critical for producing a desirable outcome in terms of the variables. The results include the environment's exposure, temperature, sunshine hour, and humidity. It would be beneficial to have a thorough understanding of the factors that contribute to “resilience” in the face of climate change in order to develop a more nuanced picture of the relationship between climate change and mental health, which would be useful when developing programmes and policies for those who are the most impacted by climate change [24].

Regarding mental health outcomes, hospital admission is the most frequently considered as the administrative data is usually available yet confidentially in the psychiatric department and can be obtained with the hospital's permission. In addition, the outcome based on the survey has some limitations, such as the issue of a survey sample that might not represent the general population.

Additionally, for the techniques used in the previous study, the researchers used the time series analysis method to identify the relationship either using statistical analysis or machine learning. However, machine learning in this domain is not widely applied where; there is only one study that used machine learning in the study. Therefore, with the recent advancement in machine learning, there is an opportunity for the researcher or computer scientist to apply the benefits of machine learning in this domain. Even some extension from machine learning (deep learning) would be an excellent technique in this domain study.

There are some limitations and research gaps that have been highlighted in the previous studies in order to improve future research.

### 5.1. Limited Sample of Data

The issue of limited sample data has been reported in a few research, for instance, a study from [30]. The consequence of limited data may reduce the performance of statistical analysis [31]. The limited number of variables used will not provide great insight into identifying the relationship between the subject matter of study. Besides, in the research using the survey in their study, they reported the issue of a survey sample that might not represent the general population.

### 5.2. Lack of Model Interpretability

Finally, the previous researchers also highlighted that causality could not be inferred from the developed model, such as mentioned by [34] that were using the regression model. Reference [36] also inferred that the correlation measures the strength between the variables but does not determine the causality. The most obvious is when nonlinearity (according to statistical tests or undetected nonlinearity) cannot be effectively captured using traditional time series models. The aforementioned limitation allows the researchers to explore further in this domain study.

## 6. Recommendation

Although prior research has examined the effects of climate change on depressive patients, knowledge gaps in this domain study still exist. For future works, it has been suggested that the researchers include more sample size, especially for studies using the survey method, to obtain a better insight from the research. Besides, selecting the variables is also crucial to conducting a good study. Future research could include more variables in the study to enrich the findings. Some variables might have complex patterns, and it may be hard to identify the relationship between climate change and depression. Therefore, it is suggested to analyze the data using a different model such as machine learning and deep learning to identify the relevant relationship. Both approaches are relatively modern and quite recent—for example, time series analysis using the long short-term memory (LSTM) model. In recent years, the application of time series using LSTM can be found in various applications, including finance, supply and demand forecasting, and health monitoring. Furthermore, the applications in a variety of disciplines have demonstrated that such methods outperform classical models [59]. While the application of machine learning and deep learning in this field of study is still limited, opportunities to explore the application of machine learning in this study are enormous.

## 7. Conclusion

This systematic review discusses the previous studies related to climate change's impact on depression. The current finding, variables, and techniques used in previous research have been demonstrated. Based on the selected articles reviewed in this SLR, there appears to be strong evidence of the association between environmental exposure related to climate change towards depressive patients. The consequences have been discussed regarding environmental exposure, mental health outcomes, and vulnerability factors. Age and gender appeared to be the most considered variable in most of the studies, with most findings on males as more vulnerable than women to climate change effects. The age of the vulnerable group varied between studies. However, the evidence is limited, and the findings vary between researchers. Therefore, more studies are needed in this domain. It is recommended that future researchers increase the sample size and use more variables to provide a better insight. The authors also recommend future research to utilize advanced technology such as machine learning or deep learning techniques to determine the relationship between climate change and depression. This domain study involves two crucial subject matters: climate change and depression, which are considered significant problems; thus, all parties should pay attention and take action for a better environmental system.

## Figures and Tables

**Figure 1:** Flow of review process adopted from [29].

**Figure 2:** Number of articles categorized by study techniques.

**Figure 3:** Publications distributed by years.

**Figure 4:** Country-wise production.

**Figure 5:** Word cloud of keywords used in the selected studies.

**Table 1:** Characteristics of the included studies.

Study	Environmental exposure	Mental health outcome	Vulnerability factors	Study techniques	Category
[30]	Temperature, humidity, hours of sunshine	Hospital admission	NA	Pearson's correlation stepwise regression	Statistical
[31]	Temperature, humidity, hours of sunshine	Hospital admission	Age, gender, residency	Log-linear function	Statistical
[32]	Temperature	Hospital admission	Age, gender	DLNM	Statistical
[33]	Hours of sunshine	Hospital admission	Age, gender	ARIMA	Statistical
[34]	Temperature, rainfall, daily hours of sunshine, duration of days	Symptom scales	Demographic, employment, urbanity, history of mental health, behavioral health, co-morbidity	Linear regression	Statistical
[35]	Temperature and water vapour	Symptom scales	Gender, age, educational attainment, relationship status, language used	Logit regression	Statistical
[36]	Temperature, atmospheric pressure, humidity, visibility, wind speed, rain, snow, storm, fog, air quality data	Symptom scales	NA	Pearson's correlation random forest, multinomial regression, support vector machine	Statistical,
					Machine learning
[37]	Temperature	Hospital admission	Age, gender, insurance amount	Cox proportional hazard	Statistical
[38]	Temperature, humidity, atmospheric pressure, rainfall, sunshine duration	Hospital admission	Age, gender, income residency, obesity, smoking status, alcohol consumption	Logistic regression	Statistical
[39]	Temperature, rainfall, daily hours of sunshine, cloudiness	Hospital admission	NA	Poisson regression	Statistical
[40]	Drought	Symptom scales	Personal income, retirement status employment status	Multivariable regression	Statistical
[41]	Drought	Symptom scales	Age, gender, ethnicity, education, income	Linear regression	Statistical
[42]	Particulate matter pollution	Hospital admission	Age, gender and season	Generalized additive model	Statistical
[43]	Air pollution	Emergency department visit	Age, gender, season, city	Logistic regression	Statistical
[44]	Air pollution, noise urban greenness	Symptom scales	Age, gender, education	Multi-exposure models	Statistical

**Table 2:** Most relevant sources.

No	Journal name	Count of papers
1	Environmental Research	2
2	Science of the Total Environment	2
3	Journal of Affective Disorders	2
4	Environmental Health Insights	1
5	BMC Public Health	1
6	BMC Research Notes	1
7	Environment International	1
8	Annals of Psychiatry and Mental Health	1
9	Psychiatry Research	1
10	PloS one	1
11	Ecohealth	1
12	International Journal of Environmental Research and Public Health	1

## Data Availability

The data used to support this systematic review are from previously reported studies, which have been cited within the manuscript.
